RETRACTED

# Clinical Characteristics and Mathematical Analysis of Curative Effect of Hemodialysis in Curing Poisoning Caused by Snakebite

**DOI:** 10.1155/2022/2312972

**Published:** 2022-05-06

**Authors:** Guoliang Huang, Bingbing Chen, Yi Luo, Liming Chen, Shaojie Wu, Shijun Wang

**Affiliations:** ^1^Department of Emergency Medicine, Emergency Medicine Department of the 910th Hospital of JLSF, Quanzhou Fujian 362000, China; ^2^Department of Emergency Medicine, Liuzhou Traditional Chinese Medical Hospital, Liuzhou Guangxi 530021, China; ^3^Fujian Provincial People Hospital, Fuzhou Fujian 350004, China

## Abstract

In order to explore the clinical characteristics of hemodialysis in curing poisoning from snakebites, a two-classification model of nuclear logistic neural network based on restricted Boltzmann machine is proposed. The model combines kernel logistic regression with artificial neural networks, enabling the model to both learn autonomously and handle linearly inseparable problems. The network first performs feature learning through unsupervised training of restricted Boltzmann machines and obtains the initial values of the parameters to be identified, which reduces the influence of the randomness of the initial parameters. The variable universe learning rate with scaling factor is used to learn the parameters to be identified, and the model convergence speed is improved by dynamic adjustment of the learning rate. Experimental results show the following: Compared with before treatment, patient's activated partial thromboplastin time (APTT) after treatment and the prothrombin time (PT) level decrease, fibrinogen (FIB) levels are elevated, aspartate transferase (AST) and creatine kinase isoenzyme (CK-MB) level decreased, and the differences were statistically significant (*p* < 0.05). It is proved that continuous hemodiafiltration combined with plasma exchange treatment can effectively improve the blood coagulation index and myocardial index of severe snakebite poisoning patients.

## 1. Introduction

Continuous renal replacement therapy is a method of extracorporeal blood purification based on hemodialysis. CRRT is hemodynamically stable and effectively removes medium and large molecules, improves inflammation, precisely controls the volume load, and adjusts the immune function and other advantages, for severe acute and chronic renal failure and its complications, acute poisoning, and heart failure, and the treatment of critical illnesses such as severe pancreatitis and crush syndrome has opened up new ways [1]. Continuous renal replacement therapy is a process that requires extracorporeal blood circulation, so the formulation of anticoagulation regimen is an important measure to ensure smooth CRRT treatment. Reasonable selection of anticoagulation regimens for blood purification is the key to ensuring and improving the success of continuous renal replacement therapy. Currently available anticoagulation methods for CRRT include the following categories: standard dose unfractionated heparin, regional citrate anticoagulation, low molecular weight heparin and heparinoid, regional heparinized anticoagulation, no anticoagulant, thrombin receptor antagonists, and platelet inhibitors, but no one anticoagulant regimen is suitable for all patients treated with CRRT, and the choice of anticoagulation regimen should be individualized. Among a variety of anticoagulants, heparin is easy to use, economical, easy to monitor, and can antagonize protamine when overdose, it is currently the most widely used anticoagulant for CRRT [2]. Heparin is an anionic sulfated mucopolysaccharide with a molecular weight of 5 kDa to 100 kDa, it forms complexes with antithrombin III in the blood, and the serine proteases of blood coagulation factors I, IX, XI, and XII lead to the rapid inactivation of these factors and plays an anticoagulant effect. The half-life of heparin in the human body is 60 min, the half-life in AKI patients is 40-180 min. The main disadvantage of heparin is that it increases the risk of bleeding and causes heparin-related thrombocytopenia [3]. At present, in the dosage of heparin, the application method and the implementation of the individualized plan are still mainly based on the experience of the clinician, various research reports differ in the dosage and implementation of CRRT heparin anticoagulation.

RETRACTED

As a classic research topic in classification problems, neural networks, in recent years, breakthrough research results have been achieved [4]. With a fast learning contrast divergence algorithm proposed by Hinton et al., and successfully applied it to deep belief network (DBN) training, the machine learning industry has set off an upsurge of research on deep learning theories and applications. The basic stacking unit of DBN restricted Boltzmann machine (RBM) is a kind of stochastic neural network and has been extensively studied [5]. Haar et al. gave the Chinese explanation of RBM, and RBM is a kind of unsupervised random neural network with two layers of visible layer and hidden layer without self-feedback and use the fast learning algorithm to unsupervised training the model [6]. Burn et al. proposed a new semisupervised learning algorithm for sentiment classification, and it is called a fuzzy deep belief network. First of all, on the training data, use semisupervised learning methods to train general DBNs, then design a fuzzy membership function, combine the previously trained DBN with the fuzzy membership function to get a new structured fuzzy DBN, and use a supervised learning algorithm to improve the classification accuracy of the model [7]. Wu et al., in order to improve the representation ability and robustness of the RBM model, proposed a new fuzzy restricted Boltzmann machine model. The weight threshold of the model connecting the visible layer and the hidden layer is taken as a fuzzy number [8]. The purpose of this study was to investigate the effect of continuous hemodiafiltration combined with plasma exchange on coagulation indexes and myocardial indexes in patients with severe snakebite poisoning. The results are reported as follows.

RETRACTED

## 2. Nuclear Logistic Neural Network Based on Restricted Boltzmann Machine

Kernel Logistic Neural Network (KLNN) combines the self-learning, self-adapting, and generalization capabilities of artificial neural networks with the processing capabilities of nonlinear features of kernel logistic regression and is superior to general kernels in structure and performance. Logistic regression technology can handle two-class and multiclass problems very well. It uses restricted Boltzmann machine to initialize the parameters of each layer of the network, which reduces the influence of randomness of parameters and avoids the model falling into the local optimum improves the overall classification accuracy of the model [9].

Suppose the input sample data set is *X* ∈ *R*^*N*×*d*^, where *N* is the number of input samples, and *d* is the feature dimension of the input sample. In the binary classification, the output vector *y* is a binary vector, for each sample input, *x*_*i*_ = [*x*_1_^*i*^, ⋯,*x*_*d*_^*i*^]^*T*^, where *i* = 1, 2, ⋯, *N* is a row vector of *X*, its corresponding output *y*_*i*_ = 1 or *y*_*i*_ = 0. Suppose the number of hidden layer nodes of the neural network is *H*, and the output node is 1.

The specific functions of each layer for any piece of input data are as follows:

The first layer is the input layer, which mainly receives sample information from the outside and passes the input vector *x*_*i*_ = [*x*_1_^*i*^, ⋯, *x*_*d*_^*i*^] directly to the next layer. The number of nodes in the input layer is the feature dimension *d* of the input sample, and the output of this layer is

(1) $$\begin{array}{c} f_{i}\left(x_{i}\right)=x_{i}. \end{array}$$

The second layer is the conversion layer, and in this layer, the kernel function is added to the input sample, that is, each node of this layer is a kernel function, the input variable passed by the input layer is transformed into *K*^0^ = *φ*(*x*_*i*_, *x*_*j*_) after kernel transformation, where *x*_*i*_ = [*x*_1_^*i*^, ⋯, *x*_*d*_^*i*^], *x*_*j*_ = [*x*_1_^*j*^, ⋯, *x*_*d*_^*j*^], *i*, *j* = 1, 2, ⋯, *N*, and *φ*(*x*_*i*_, *x*_*j*_) is the conversion function, and *K*^0^ ∈ *R*^*N*×*N*^ is the input signal after adding the kernel function, it can be expressed as the following form:

(2) $$\begin{array}{c} K^{0}=\left[\begin{array}{cccc} k_{11}^{0} & k_{12}^{0} & \cdots & k_{1N}^{0}\\ k_{21}^{0} & k_{22}^{0} & \cdots & k_{2N}^{0}\\ \cdots & \cdots & \cdots & \cdots \\ k_{N1}^{0} & k_{N2}^{0} & \cdots & k_{NN}^{0} \end{array}\right]={\left[k_{1}^{0},k_{2}^{0},\cdots ,k_{N}^{0}\right]}^{T}, \end{array}$$

where *k*_*i*_^0^ = [*k*_*i*1_^0^, *k*_*i*2_^0^, ⋯,*k*_iN_^0^]^*T*^ is line *i* of *K*^0^, *i* = 1, 2, ⋯, *N*. There are many forms of conversion function when selecting, using linear kernel function and Gaussian kernel function.

RETRACTED

As the addition of the kernel function makes the structure of the model more complicated, the introduction of high dimensions increases the noise of the data, and in order to reduce the amount of calculation, the principal component analysis (PCA) method is used to reduce the dimensionality of the input sample data of this layer, the first *n* principal components are selected as the output of the conversion layer [10].

After dimensionality reduction by PCA algorithm, new output sample data *K* ∈ *R*^*N*×*n*^ is obtained, where *n* is the dimension of the kernel matrix after dimensionality reduction, and the kernel matrix can be expressed as

(3) $$\begin{array}{c} K=\left[\begin{array}{cccc} k_{11} & k_{12} & \cdots & k_{1n}\\ k_{21} & k_{22} & \cdots & k_{2n}\\ \cdots & \cdots & \cdots & \cdots \\ k_{N1} & k_{N2} & \cdots & k_{Nn} \end{array}\right]={\left[k_{1},k_{2},\cdots ,k_{N}\right]}^{T}, \end{array}$$

where *k*_*i*_ = [*k*_*i*1_, *k*_*i*2_, ⋯,*k*_in_]^*T*^ is line *i* of *K*, *i* = 1, 2, ⋯, *N*. The output of this conversion layer can be expressed as

(4) $$\begin{array}{c} f_{2}\left(x_{i}\right)=PCA\left(\varphi \left(x_{i},x_{j}\right)\right)=k_{i}. \end{array}$$

The third layer is the hidden layer, receive the sample information after principal component analysis dimensionality reduction and pass it to the logistic regression layer. Suppose the number of neurons in this layer is *H*, connection weights and thresholds are *ω*_*h*_, and *θ*, *ω*_*h*_ ∈ *R*^*n*×*H*^, is a matrix of *n* × *H*, *θ* ∈ *R*^*H*×1^, is a vector of *H* × 1. Enter the value *k*_*i*_ = [*k*_*i*1_, ⋯,*k*_in_]^*T*^, *i* = 1, 2, ⋯, *N*, for each sample of this layer, and the corresponding output value *G*_*i*_ is expressed as

(5) $$\begin{array}{c} G_{i}=\sigma \left(\theta +\overset{n}{\underset{j=1}{\sum }}\omega_{jh}\cdot k_{ij}\right)=\sigma \left(\theta +\omega_{h}^{T}\cdot k_{i}\right). \end{array}$$

For the activation function of the hidden layer, we take the Sigmoid function, and the output value of the *σ*(*u*) = 1/1 + *e*^−*u*^ hidden layer can be expressed as

(6) $$\begin{array}{c} f_{3}\left(k_{i}\right)=G_{i}=\frac{1}{1+e^{-\left(\theta +\omega_{h}^{T}\cdot k_{i}\right)}}. \end{array}$$

The fourth layer is the logistic regression layer, and the logistic function is used to calculate the output information of the hidden layer. The input information of this layer is a vector *G*_*i*_ of *H* × 1, the logistic regression parameter and threshold are *β*, *α*, respectively. Where *β* ∈ *R*^*H*×1^ is a column vector of *H* × 1, and *θ* is a constant. For two classifications, the probability formula for *y*_*i*_ = 1 can be obtained, that is, the logistic function:

(7) $$\begin{array}{c} P_{i}=P_{i}\left(y_{i}=1\right)=\sigma \left(\alpha +\overset{H}{\underset{h=1}{\sum }}\beta_{h}\cdot \sigma \left(\theta +\omega_{h}\cdot k_{i}\right)\right)=\sigma \left(\alpha +\overset{H}{\underset{h=1}{\sum }}\beta_{h}\cdot G_{i}\right) \end{array}$$

From this, the probability formula for *y*_*i*_ = 0 can also be obtained:

(8) $$\begin{array}{c} P_{i}\left(y_{i}=0\right)=1-P_{i}\left(y_{i}=1\right)=1-\sigma \left(\alpha +\overset{H}{\underset{h=1}{\sum }}\beta_{h}\cdot G_{i}\right). \end{array}$$

For formula (7), take *σ*(*u*) = 1/1 + *e*^−*u*^, so the output value of the logistic regression layer can be expressed as

(9) $$\begin{array}{c} f_{4}=P_{i}=\sigma \left(\alpha +\overset{H}{\underset{h=1}{\sum }}\beta_{h}\cdot \sigma \left(\theta +\omega_{h}\cdot k_{1}\right)\right)=\sigma \left(\alpha +\overset{H}{\underset{h=1}{\sum }}\beta_{h}\cdot G_{i}\right)=\frac{e^{\beta^{T}\cdot G_{i}+\alpha }}{1+e^{\beta^{T}\cdot G_{i}+\alpha }}. \end{array}$$

The fifth layer is the output layer, and the output of the binary classification can be defined as

(10) $$\begin{array}{c} f_{5}=y_{i}=\left\{\begin{array}{cc} 1,\text{if} & P_{i}\geq 0.5,\\ 0,\text{if} & P_{i}<0.5. \end{array}\right. \end{array}$$

It can be seen from the binary classification model of the nuclear logistic neural network that the parameters that need to be optimized are the connection weight *ω*_*h*_ and threshold *θ* of the hidden layer and the regression parameter *β* and threshold *α* of the logistic regression layer. The following explains how to identify the parameters of the model. The KLNN-RBM learning algorithm is proposed to identify the parameters of the nuclear logistic neural network. The basic process of the algorithm is as follows: The restricted Boltzmann machine is used for unsupervised training of the initial weights and thresholds of the nuclear logistic neural network regression model, get the optimal initial value of the model parameters, and add the ridge regression regularization factor to the log-likelihood function in the logistic regression layer to estimate the maximum likelihood. On this basis, we use the stochastic gradient descent method with variable universe expansion factor to train the model parameters, by dynamically adjusting the learning rate to change the speed of training, improving the overall classification accuracy of the model [11].

RETRACTED

## 3. Simulation Experiment

We selected 30 cases of severe snakebite poisoning patients who were admitted to a hospital from January 2019 to October 2020 and all meet the selection criteria: (1) inclusion criteria were as follows: ① meet the diagnostic criteria for severe snakebite poisoning; ② all were admitted to the hospital for treatment within 48 hours after being bitten; ③ this study was approved by the medical ethics committee, and the patient was informed of this study and signed a consent form; and ④ there is no contraindication to treatment. (2) exclusion criteria were as follows: ① patients with other blood system diseases; ② patients with damage to the heart, liver, and other organs; and ③ patients with coagulation dysfunction. Among the 30 patients, there were 17 males and 13 females; age ranged from 28 to 52 years old, with an average of39.69 ± 7.03years old. Snake species are as follows: 10 cases were bitten by Bamboo Leaf Green snake, 9 cases were bitten by silver ring snake, and 9 cases were bitten by cobra 11 cases; bite site is as follows: 11 cases of hand and arm, 13 cases of foot, and 6 cases of lower extremity. The local area of the bite was markedly swollen, and ecchymosis was visible under the skin, and the pain was severe. The data collected for each sample covers 19 physiological indicators, such as the patient's gender, age, creatinine, albumin, hemoglobin, and survival time, and among them, the gender of the patient, whether the circulatory system has heart failure, whether the digestive system has nausea and vomiting, whether there is edema in the urinary system, whether the endocrine system suffers from diabetic nephropathy, six indicators, such as whether the nervous system suffers from uremic encephalopathy, are binary data, and the other 13 indicators are numerical data [12].

### 3.1. Conventional Treatment

After the patient was admitted to the hospital, the wound exudate, blood, etc. were detected by enzyme-linked immunosorbent assay from the patients who were bitten by an unknown species of snake to confirm the specie of the venomous snake. At the same time, conventional treatment was given, the wound was swollen and compressed with a bandage, the wound was debridement locally, and the corresponding antivenom serum was injected according to the type of venomous snake to stop bleeding, infection, etc. and the patient was instructed to keep quiet and not to panic to prevent the spread of the venom [13].

RETRACTED

### 3.2. Continuous Hemodiafiltration Combined with Plasma Exchange Therapy

#### 3.2.1. Plasma Exchange Treatment

For the application of plasma separator, use indwelling internal jugular vein or femoral vein catheter to establish vascular access and aseptically install extracorporeal circulation pipelines and plasma separators as required. First, flush the pipeline with saline, then rinse with 0.2 g/L heparin saline, and when the blood flow rate is 120 ml/min, choose 2500~3000 ml of fresh plasma and human albumin solution as the replacement fluid, replace once every 2.5 to 3 hours and once a day.

#### 3.2.2. Continuous Hemodiafiltration Treatment

For continuous hemodiafiltration treatment, use the hemodialysis machine, select the continuous venous hemodiafiltration mode, establish a vascular access in the patient's central venous catheter, control the blood flow rate to 180 ml/min, adjust the temperature of the dialysate to 35~35.5°C, while drawing blood, instill 150 ml and 50% glucose solution at 20-30 drops/min. Decide whether to pump heparin for anticoagulation treatment according to the patient's condition, hemodiafiltration was performed 1 to 2 times, and each treatment was performed for 24 to 48 hours. After treatment, the patient's condition was stable and his vital signs were normal [14].

Since the collected sample data contains more indicator information, how to determine the key indicators that affect the relationship between dialysis timing and patient survival time, it is the main problem that needs to be solved. The proposed nuclear logistic neural network model based on the restricted Boltzmann machine analyzes the modeling data, and the classification results are used to mine the index variables used to establish the hemodialysis evaluation model. This section uses the training data set from 2019 to 2020 for analysis. The main input variables considered included patient's gender (Gen), patient's age at first dialysis (age), creatinine (Scr), albumin (Alb), urea (BUN), hemoglobin (Hb), serum phosphorus (P), serum potassium (K), heart failure (HF), diabetes (DM), nausea and vomiting (DIG), edema (URI), and uremic encephalopathy (NEU). The main consideration is based on the first 5 attributes, find the best combination of variables that affect the timing of hemodialysis. The output index is the survival time of the patient from the first dialysis, it is measured on a monthly basis. Figures 1–4, respectively, show the distribution line graphs of 4 numerical indicators [4, 15–17].

RETRACTED

## 4. Results and Analysis

### 4.1. Comparison of Coagulation Indexes before and after Treatment

Compared with before treatment, the APTT and PT levels of patients after treatment are reduced, FIB levels increased, and the differences were statistically significant (*p* < 0.05). See Table 1.

### 4.2. Comparison of Myocardial Indexes before and after Treatment

Compared with before treatment, the AST and CK-MB levels of the patients after treatment decreased, and the difference was statistically significant (all *p* < 0.05). See Table 2.

## 5. Discussion

There are many kinds of snakes, cobras, green bamboo leaves, etc. are all common species; therefore, epidemiology shows that the fatality rate and disability rate of poisonous snakebites are relatively high. Due to the large molecular proteins contained in snake venom, toxic substances such as small peptides quickly enter the bloodstream and can cause symptoms of systemic poisoning, and if not treated in time, it can cause damage to human liver and kidney function, even life-threatening. At present, the main principle of treating snakebite is to block the spread of snake venom in the body, to eliminate its harmful toxins, and to protect the function of important organs. Studies have shown that early treatment measures can effectively save the lives of patients.

The liver is the main organ for the body to synthesize blood clotting factors, and it plays a role in maintaining balance in the coagulation and anticoagulation system. After being bitten by a poisonous snake, snake venom entering the body can cause severe symptoms of poisoning, lead to damage to liver function, which in turn leads to a decrease in coagulation factors, abnormal blood clotting function. Clinical detection of elevated levels of AST and CK-MB indicators indicates that there is damage to liver cells or cardiomyocytes, so it is of great significance to detect coagulation indicators and myocardial indicators in patients with snakebite. The results of this study showed that compared with before treatment, the levels of APTT, PT, AST, and CK-MB in patients after treatment were decreased, and the level of FIB was increased, suggesting that continuous hemodiafiltration combined with plasma exchange therapy can effectively improve severe snakebite. Coagulation indexes and myocardial indexes of patients with trauma and poisoning analyze the reasons and believe that plasma exchange is a kind of extracorporeal circulation blood purification therapy, and its working principle is by drawing the patient's whole blood out of the body, separate plasma and cell components, discard the patient's plasma, then replace fresh plasma, albumin, and other substitutes at the same speed, back into the body, ultimately achieve the purpose of reducing disease damage. Since snake toxin enters the body, it can be combined with protein, blood lipids, etc. or dissolved in the plasma; plasma exchange can remove the poisonous substances from snake venom in the body in time, and at the same time, supplementation of coagulation factors can quickly play a role in the body, and the earlier the treatment, the more obvious the effect, conducive to improve the success rate of rescue and improve the clinical symptoms of patients bitten by poisonous snakes. Plasma exchange is used to treat venomous snakebites and can quickly remove toxins, improve the patient's blood hypercoagulability state, and improve the success rate of treatment. And the incidence of plasma exchange complications is relatively small, common complications are mainly related to abnormalities in the patient's cardiopulmonary bypass, and fresh plasma is not related to factors such as discomfort and it can cause adverse reactions such as infection, bleeding, and hypotension [18]. Continuous hemodiafiltration can effectively maintain the body's water and electrolyte stability, remove toxins in the circulation, improve the nutritional status of patients, and facilitate the restoration of damaged cells; at the same time, it can promote hemodynamic stability and it is beneficial to maintain the body environment, to promote the recovery of patients and improve the survival rate [19]. Continuous hemodiafiltration combined with plasma exchange in the treatment of severe snakebite patients can play a synergistic effect, alleviate the insufficiency of single treatment, effectively remove snake toxins, improve blood coagulation and myocardial indicators, improve the success rate of treatment, and reduce the risk of death of patients. However, due to the small sample size, this study has certain limitations, and it is necessary to further increase the sample size to demonstrate the feasibility of this treatment plan.

RETRACTED

## 6. Conclusion

A two-classification model and a multiclassification model of nuclear logistic neural network based on restricted Boltzmann machine are proposed. In the binary classification model of the nuclear logistic neural network, the input data is mapped from the low-dimensional feature space to the high-dimensional through a kernel function, solve the linear inseparability problem, and through principal component analysis to reduce the dimensionality of the data, avoid the amount of calculation caused by nuclear transformation. The network initializes the weights and thresholds of each layer through unsupervised learning RBM, it greatly improves the classification accuracy of the overall model; to reduce the influence of random parameters, the log-likelihood function with ridge regression regular term is used as the objective function for maximum likelihood estimation, and redundant features are eliminated to avoid overfitting. In snakebite, in addition to the acute renal failure caused by dialysis treatment, other system damage using dialysis treatment has not been reported, and the mechanism is unknown. In this group of cases, there were complications, such as respiratory failure, shock, heart failure, and renal failure, all of which were cured after conventional treatment. Therefore, we believe that dialysis has a definite effect on snakebite.

## Figures and Tables

**Figure 1:** Line chart of the distribution of albumin index.

**Figure 2:** Line chart of the distribution of leucin indicators.

**Figure 3:** Broken line chart of the age distribution of patients on dialysis.

**Figure 4:** Line chart of the distribution of blood phosphorus indicators.

**Table 1:** Comparison of coagulation indexes before and after treatment.

Project	APTT	FIB	PT
Before therapy	44.67 ± 3.55	0.91 ± 0.46	18.29 ± 3.44
After treatment	29.61 ± 2.44	3.20 ± 0.68	10.06 ± 1.15
*t* value	30.953	15.724	21.040
*p* value	*p* ≤ 0.001	*p* ≤ 0.001	*p* ≤ 0.001

**Table 2:** Comparison of myocardial indexes before and after treatment.

Project	AST	CK-MB
Before therapy	70.95 ± 12.58	49.49 ± 10.27
After treatment	21.52 ± 2.43	18.57 ± 2.63
*t* value	32.247	24.625
*p* value	*p* ≤ 0.001	*p* ≤ 0.001

## Data Availability

The data used to support the findings of this study are available from the corresponding author upon request.
